The article "The Accuracy of 16S rRNA Polymerase Chain Reaction for the Diagnosis of Neonatal Sepsis: A Meta-Analysis" was published in 2021. Journal: Biomed Res Int.

# The Accuracy of 16S rRNA Polymerase Chain Reaction for the Diagnosis of Neonatal Sepsis: A Meta-Analysis

**DOI:** 10.1155/2021/5550387

**Published:** 2021-05-12

**Authors:** Ying Wang, Jingyi Zhao, Yinhui Yao, Lan Yang, Dan Zhao, Shiquan Liu

**Affiliations:** ^1^Department of Pharmacy, The Affiliated Hospital of Chengde Medical College, Chengde 067000, China; ^2^Department of Functional Center, Chengde Medical College, Chengde 067000, China; ^3^Institute of Chinese Materia Medica, Chengde Medical College, Chengde 067000, China; ^4^Department of Intensive Care Unit, The Affiliated Hospital of Chengde Medical College, Chengde 067000, China; ^5^Department of Thoracic Surgery, The Affiliated Hospital of Chengde Medical College, Chengde 067000, China

## Abstract

**Objective:**

To determine the accuracy of 16S rRNA polymerase chain reaction (PCR) for the diagnosis of neonatal sepsis through a systematic review and meta-analysis.

**Methods:**

Studies involving 16S rRNA PCR tests for the diagnosis of neonatal sepsis were searched in the PubMed, Medline, Embase, and Cochrane Library databases. The methodological quality of the identified studies was evaluated using the Quality Assessment of Diagnostic Accuracy Studies-2 (QUADAS-2), and the sensitivity, the specificity, the positive likelihood ratio (PLR), the negative likelihood ratio (NLR), the diagnostic odds ratio (DOR), and the area under the curve (AUC) of operator characteristic (SROC) curves were determined. Heterogeneity between studies was analyzed by metaregression. Stata 14.0 and Meta-disc 1.4 software were used for the analyses.

**Results:**

This meta-analysis included 19 related studies. The analysis found a sensitivity of 0.98 (95% CI: 0.85-1), specificity of 0.94 (95% CI: 0.87-0.97), PLR of 16.0 (95% CI: 7.6-33.9), NLR of 0.02 (95% CI: 0.00-0.18), DOR of 674 (95% CI: 89-5100), and AUC of 0.99 (95% CI: 0.97-0.99). Metaregression analysis identified Asian countries, arterial blood in blood samples, and sample size > 200 as the main sources of heterogeneity. This meta-analysis did not uncover publication bias. Sensitivity analysis showed that the study was robust. Fagan's nomogram results showed clinical usability.

**Conclusions:**

The results from this meta-analysis indicate that 16S rRNA PCR testing is effective for the rapid diagnosis of neonatal sepsis.

## 1. Introduction

Neonatal sepsis, a systemic inflammatory reaction to the invasion of bacteria, viruses, fungi, and other pathogens in a newborn's blood, produces toxins and is the most common form of infectious disease among newborns [1]. Globally, neonatal sepsis has an intimate connection with a 2.2% morbidity rate and a mortality rate of 11-19%, with higher mortality in developing countries [2, 3]. Clinical signs of neonatal sepsis are often aspecific, which limits initial diagnosis. Late diagnosis leads to disease progression, resulting in multiple organ failure and even death. Thus, early diagnosis of sepsis and early treatment are key to successful outcomes.

The gold standard for the diagnosis of neonatal sepsis is through culture of the microorganisms from patient blood or other body fluids, such as urine, and cerebrospinal fluid. However, due to factors such as insufficient samples, maternal use of antibiotics, and antibiotic use before sampling, this method may give false negative results [4, 5]. Various biomarkers, including C-reactive protein (CRP), procalcitonin (PCT), neutrophil CD64, interleukin-8, and interleukin-27, are used for sepsis diagnosis [6–11]. However, these biomarkers may also be elevated in noninfectious conditions such as premature rupture of membranes, fetal distress, dystocia, and perinatal asphyxia, resulting in false positive results and low specificity for neonatal sepsis [6]. Thus, there is an urgent need for faster, more sensitive tests for neonatal sepsis diagnosis.

Recently, the PCR technique has been universal deployed in clinical diagnoses, which makes it possible to diagnose infectious diseases caused by microorganisms quickly and accurately. Moreover, numerous studies have shown that 16S rRNA PCR can diagnose neonatal sepsis [12–17]. The 16S rRNA gene is 1500 nucleotides long and encodes the 30S ribosomal subunit in all prokaryotes. The 16S rRNA gene is highly conserved and does not change over time. Within a certain range, the 16S rRNA gene can accurately identify specific bacteria based on gene-specific signatures [18, 19]. Relative to culture techniques, 16S rRNA PCR is cost-effective and rapid [20]. Here, we conducted a systematic review and meta-analysis of published studies to determine the utility of 16S rRNA PCR in neonatal sepsis diagnosis.

## 2. Methods

### 2.1. Search Strategy

Two authors independently performed literature searches of PubMed, Medline, Embase, and the Cochrane Library using the search terms 16S rRNA, 16S ribosomal ribonucleic acid, septic, septicemia, and neonatal sepsis. No restrictions were applied on the search, which included studies published until 13 January 2021. To ensure comprehensive literature identification, we manually searched relevant references in the identified studies.

### 2.2. Study Selection

The following inclusion criteria were used: (1) samples were neonatal blood; (2) true positive (TP), true negative (TN), false positive (FP), and false negative (FN) values could be directly or indirectly obtained; (3) all data were derived from 16S rRNA PCR tests for neonatal sepsis diagnosis. The exclusion criteria were as follows: (1) literature in the form of review, meta-analysis, case report, or letter; (2) studies that were not clearly defined as involving neonates; (3) studies in with insufficient data for meta-analysis; and (4) studies involving nonblood samples.

### 2.3. Data Extraction

The following data were extracted by 2 authors: first author name, publication year, region, TN, FN, TP, FP, test method, and test sample. Disagreements were resolved by a 3^rd^ author.

### 2.4. Quality Assessment

The inclusion criteria and methodological quality of selected articles were evaluated by 2 independent authors using QUADAS-2 [21], and disagreements were resolved by a 3^rd^ author.

### 2.5. Statistical Analysis

Study heterogeneity was evaluated by *I*^2^ test. Heterogeneity due to the threshold effect was evaluated by the Spearman model. When study heterogeneity was statistically significant (*I*^2^ > = 50% or *p* = <0.05), the random effect model was used; otherwise, a fixed effects model was used [22, 23]. To evaluate 16S rRNA PCR potential and accuracy in neonatal sepsis diagnosis, sensitivity, specificity, PLR, NLR, DOR, and AUC of SROC curve analyses were used. Metaregression analysis was used to determine heterogeneity sources. Deeks' funnel plot asymmetry test was used to evaluate publication bias [24]. Sensitivity analysis was used to evaluate the robustness of this study. Statistical analyses were performed by Stata 14.0 and Meta-disc 1.4.

## 3. Results

### 3.1. Study Characteristics

A total of 2545 studies were identified, and 1058 duplicate studies were eliminated. Upon title and abstract review, 1368 studies were excluded, and 119 were subjected to full-text review. Of these, 100 were excluded because valid data could not be extracted, and the remaining 19 articles were included in our study [12, 13, 25–41] (Figure 1).

The19 articles incorporated into in our study involved a comparison between the diagnostic value of 16S rRNA PCR and blood culture for pathogenic microorganism identification in neonatal sepsis patients. The important features of the 19 articles are displayed in Table 1. They involved a total of 4740 neonatal blood samples, of which 553 were positive and 4187 were negative. The included studies were from Turkey (1), China (6), Egypt (3), India (4), Israel (1), the US (1), Japan (1), Italy (1), and Sweden (1). 16S rRNA amplification was achieved by PCR.

### 3.2. Quality Assessment

Methodological quality and risk of bias in the included studies were assessed using QUADAS-2. All studies used a prospective study design to avoid inappropriate exclusion (Figure 2). Five studies did not specify whether patients were continuously enrolled or not [25, 26, 28–30]. The remaining studies specified continuous enrollment. The reference standard in all studies was pathogenic microorganism blood culture. Some studies did not report sufficient data on indicator tests and/or reference criteria, so these items were used as ambiguous risk of bias scores. QUADAS-2 did not include an overall bias score, but the overall quality of the studies included in the analysis was moderate to high.

### 3.3. Heterogeneity Analysis and Diagnostic Accuracy

The sensitivity *I*^2^ was 99.95 (95% CI: 99.94-99.55), *p* ≤ 0.001. And the specificity *I*^2^ was 99.32 (95% CI: 99.23-99.42), *p* ≤ 0.001. Because the results point out heterogeneity among the studies, the random effect model was adopted. Analysis results were displayed in Figure 3. The overall sensitivity and specificity of the 19 studies were 0.98 (95% CI: 0.85-1.00) and 0.94 (95% CI: 0.87-0.97), respectively. The PLR was 16.0 (95% CI: 7.6-33.9), the NLR was 0.02 (95% CI: 0.00-0.18), and the DOR was 674 (95% CI: 89-5100). The SROC curve analysis of the 16S rRNA gene PCR test accuracy in neonatal sepsis diagnosis revealed an AUC of 0.99 (95% CI: 0.97-0.99; Figure 4).

### 3.4. Subgroup Analysis and Metaregression

In order to investigate the potential sources of heterogeneity, we conducted threshold effect analysis using Meta-disc 1.4 and obtained a Spearman correlation coefficient of 0.262 (*p* = 0.279), indicating that the threshold effect was not the source of the heterogeneity. Next, metaregression analysis was used to divide the subgroups into location (Asian vs. non-Asian), specimen (arterial vs. nonarterial blood), center (single center vs. multicenter), and sample size (≥200 vs. <200) (Figure 5). The main sources of sensitivity heterogeneity were location, specimen, center, and sample size. Specificity heterogeneity was mainly due to sample size.

### 3.5. Sensitivity Analysis

Sensitivity analysis was used to evaluate the reliability and robustness of the analysis results. The validity and robustness of the models involved in the statistical analyses were verified by goodness-of-fit and bivariate normality analysis (Figures 6(a) and 6(b)). Influence analysis (Figure 6(c)) showed 3 influence studies, and outlier detection (Figure 6(d)) found 1 outlier study. Sequential exclusion of influencing factors and outliers did not significantly alter the overall results (Table 2).

### 3.6. Clinical Utility of the Index Test

To evaluate posttest probabilities, Fagan's nomogram could be used to calculate the posttest probability of 16S rRNA PCR for neonatal sepsis diagnosis. When the pretest probability was set at 11%, it was found that the probability of neonatal sepsis was 0.66 if the results were positive and 0 if the results were negative (Figure 7). A likelihood ratio scatter plot showed that 16S rRNA PCR was effective for neonatal sepsis diagnosis (positive) and exclusion (negative), with the summary point of the probability ratio in the upper left quadrant (Figure 8).

### 3.7. Publication Bias

Deeks' funnel plot asymmetry test on the 19 included studies found no publication bias (Figure 9, *p* = 0.09).

## 4. Discussion

Past studies demonstrated the high potential of 16S rRNA PCR tests for diagnosing bloodstream infections. This strategy has been suggested to be effective and fast for screening sepsis [42]. In this meta-analysis, we evaluated the performance of 16S rRNA PCR for neonatal sepsis diagnosis relative to blood culture techniques. 16S rRNA PCR tests have the potential to accelerate neonatal sepsis diagnosis, thereby ensuring timely and effective treatment.

Our analysis found that the sensitivity and specificity of 16S rRNA PCR tests for neonatal sepsis diagnosis were 0.98 (95% CI: 0.85-1.00) and 0.94 (95% CI: 0.87-0.97), respectively, indicating high diagnostic effectiveness. The SROC curve showed the trade-off between the sensitivity and specificity of diagnostic research, and the AUC of the SROC curve is a measure of the integrity of the diagnostic testing ability, providing a precise basis for the overall study [43]. Our analysis revealed an AUC of 0.99 (95% CI: 0.97-0.99), indicating that 16S rRNA PCR is highly accurate for neonatal sepsis diagnosis. The DOR is a way of the usefulness of a diagnostic test and is given as a value between 0 and ∞, and a higher value means better performance. Conversely, a value of <1 indicates that the test lacks the ability to distinguish between outcomes [44]. Our analysis revealed a DOR value of 674 (95% CI: 89-5100), indicating high accuracy. The likelihood ratio fully reflects the diagnostic value of a screening test and is very stable. The DOR comprises the PLR (ratio of true positive rate to false positive rate, where the larger the ratio is, the greater the likelihood of a true positive test result) and the NLR (ratio of false negative rate to true negative rate, where the smaller the ratio is, the greater the chance of a true negative test result). Our pooled results revealed a PLR of 16.0 (95% CI: 7.6-33.9) and NLR of 0.02 (95% CI: 0.00-0.18), indicating that 16S rRNA PCR has good diagnostic ability.

Although the 16S rRNA PCR test was effective, there was significant heterogeneity in this meta-analysis. Different regions were also major sources of heterogeneity in this study. In the Asian population relative to the non-Asian populations, the sensitivity, specificity, PLR, NLR, DOR, and AUC were 1.00 (0.89-1.00) vs. 0.71 (0.41-0.89), 0.91 (0.79-0.97) vs. 0.96 (0.89-0.98), 11.5 (4.4-30.3) vs. 16.7 (7.0-39.5), 0 (0-0.14) vs. 0.31 (0.13-0.72), 4297 (64-289895) vs. 55 (17-180), and 1.00 (0.99-1.00) vs. 0.95 (0.93-0.97), respectively. Blood sample sources, sample sizes, and single- or multicenter studies were also sources of heterogeneity. However, because there were few multicenter studies, more standardized multicenter studies are needed to better understand the value of 16S rRNA PCR tests in neonatal sepsis diagnosis [45].

Our meta-analysis has some limitations. First, the included studies defined sepsis using different criteria, which may be reflected in different clinical symptoms and routine blood tests for the included patients. Although blood culture, the gold standard for sepsis diagnosis, was used in all studies, the associated false positive rate was high [4]. Second, the kits and testing tools used for blood cultures and testing were manufactured by different companies, and there are no studies on whether the results vary by kit manufacturer. Third, most studies included in this meta-analysis did not distinguish between early-onset sepsis and late-onset sepsis. Thus, we could not carry out subgroup analysis between early-onset sepsis and late-onset sepsis.

## 5. Conclusions

In summary, this meta-analysis shows that 16S rRNA PCR tests are effective for rapid neonatal sepsis diagnosis. However, PCR amplification methods are not fully defined, and future prospective studies should carry out subgroup analysis of PCR methods.

## Figures and Tables

**Figure 1:** Study selection flow chart.

**Figure 2:** Risk of bias and applicability concerns in the included studies.

**Figure 3:** Forest plots for pooled sensitivity and specificity of neonatal sepsis diagnosis by 16S rRNA PCR.

**Figure 4:** 16S rRNA symmetrical summary receiver operator characteristic (SROC) curve for all 19 studies.

**Figure 5:** Univariable metaregression and subgroup analyses.

**Figure 6:** Stability and robustness analysis of the included studies.

**Figure 7:** Fagan's nomogram for calculating the post-test probabilities of 16S rRNA PCR for neonatal sepsis diagnosis.

**Figure 8:** Likelihood ratio scatter gram.

**Figure 9:** Deeks' funnel plot for identifying publication bias.

**Table 1:** The important features of the 19 articles included in this meta-analysis.

Author	Year	Country	TP	TN	FN	FP	Specimen	Center	Threshold
İstanbullu K [25]	2019	Turkey	1	2	5	92	Blood	Single	Florescence
EL-Amir [26]	2019	Egypt	51	0	13	11	Venous	Single	380 base pairs and 212
Yu R [12]	2020	China	31	25	0	4	Blood	Single	1380 bp
Punia H [27]	2017	India	66	3	0	31	Blood	Single	203 bp
Midan DA [28]	2016	Egypt	28	4	0	8	Intravenous	Single	Fluorescent sensor
Rohit A [29]	2016	India	28	27	6	36	Peripheral	Single	996 bp
El Gawhary S [30]	2015	Egypt	10	6	6	40	Peripheral	Single	200 bp
Dutta S [31]	2009	India	50	7	2	183	Blood	Single	380 bp
Liu CL [32]	2014	China	95	28	0	583	Venous	Multicenter	630 and 216 bp
Fujimori M [33]	2010	Japan	6	9	0	24	Arterial	Single	NA
Ohlin A [34]	2008	Sweden	21	12	29	233	Intravenous	Single	CP value with a range
Wu YD [35]	2007	China	20	23	0	787	Venous	Single	CT values ≤ 35 cycles
Jordan JA [36]	2006	USA	7	30	10	1186	Venous	Single	380 bp
Makhoul IR [37]	2005	Israel	9	0	4	202	Venous	Single	997 bp
Shang S [38]	2005	China	8	9	0	155	Venous	Single	371 bp
Yadav AK [13]	2005	India	9	4	0	87	Venous	Single	861 bp
Tong MQ [39]	2004	China	8	9	0	268	Venous	Single	371 bp
Shang S [40]	2001	China	26	0	0	30	Blood & CFS	Single	371 bp
Laforgia N [41]	1997	Italy	4	2	0	27	Venous	Single	861 bp

**Table 2:** Summary estimates of the diagnostic performance of 16S rRNA PCR in neonatal sepsis diagnosis.

Analysis	Number of studies	Sensitivity (95% CI)	Specificity (95% CI)	PLR (95% CI)	NLR (95% CI)	DOR (95% CI)	AUC (95% CI)
Overall	19^12, 13, 25-41^	0.98 (0.85-1.00)	0.94 (0.87-0.97)	16.0 (7.6-33.9)	0.02 (0.00-0.18)	674 (89-5100)	0.99 (0.97-0.99)
Influence studies excluded	16^13, 25-28, 30-36, 38-41^	0.99 (0.84-1.00)	0.95 (0.92-0.97)	19.5 (12.9-29.4)	0.01 (0.00-0.20)	1464 (103-20881)	0.98 (0.96-0.99)
Outlier excluded	18^13, 25-41^	0.97 (0.83-1.00)	0.95 (0.91-0.97)	19.2 (10.6-34.7)	0.03 (0.00-0.20)	612 (87-4290)	0.98 (0.97-0.99)

## Data Availability

The data of Table 1 used to support the findings of this study are included within the article (see References).
